# An Enhanced Priori Knowledge GAN for CT Images Generation of Early Lung Nodules with Small-Size Labelled Samples

This article has been retracted.

**DOI:** 10.1155/2022/2129303

**Published:** 2022-06-14

**Authors:** Xun Wang, Zhiyong Yu, Lisheng Wang, Pan Zheng

**Affiliations:** ^1^College of Computer Science and Technology, China University of Petroleum (East China), Qingdao 266580, China; ^2^University of Canterbury, Christchurch 8140, New Zealand

## Abstract

The small size of labelled samples is one of the challenging problems in identifying early lung nodules from CT images using deep learning methods. Recent literature on the topic shows that deep convolutional generative adversarial network (DCGAN) has been used in medical data synthesis and gained some success, but does not demonstrate satisfactory results in synthesizing CT images. It primarily suffers from the problem of model convergence and is prone to mode collapse. In this paper, we propose a generative adversarial network (GAN) model with prior knowledge to generate CT images of early lung nodules from a small-size of labelled samples, i.e., SLS-PriGAN. Particularly, a knowledge acquisition network and a sharpening network are designed for priori knowledge learning and acquisition, and then, a GAN model is developed to produce CT images of early lung nodules. To validate our method, a general fast R-CNN network is trained using the CT images generated by SLS-PriGAN. The experiment result shows that it achieved a recognizing accuracy of 91%, a recall rate of 81%, and *F*1 score of 0.85 in identifying clinic CT images of early lung nodules. This provides a promising way of identifying early lung nodules from CT images using deep learning with small-size labelled samples.

## 1. Introduction

Neural networks, particularly deep learning models, have shown promising results in the field of cancer-targeted detection. Some studies have shown the ability of trained neural network models can reach the level of human physicians in lesion detection [1–4]. Almost all the methods are based on training with a large volume of datasets, which would fail when the amount of data is sparse and lacking [5, 6].

The small size of labelled samples has become one of the challenging problems in identifying early lung nodules from CT Images using deep learning technology. When there are a small number of patients screened for early pulmonary nodules, it is difficult to develop large datasets of CT images for the purpose of machine learning methods and model developments. It is formulated in [5, 7] that the small size of labelled samples has become a natural barrier to the use of neural network models in medical imaging.

A common solution to this problem is to design data synthesis methods. A typical one is to process the data set image by using translation, rotation, flip, and zoom to achieve data augmentation. Such a method has some drawbacks. Due to their inherent characteristics, medical images tend to lose their original interpretation during the process. Moreover, it is difficult to add additional useful information to the dataset for the training of neural network algorithms. Usually, the datasets used by these networks have both input and expected output, and the difference between the generated and the expected output is defined as the loss function [8–11]. It is shown in [10] that when the original data is lost or unavailable, the generated images can be used to diagnose Alzheimer's disease. This kind of model requires a large amount of data for training, and the performance of the network model on a small set of sample data is less accurate and sufficient.

Generative adversarial networks (GAN), which have a generator and a discriminator, are used to do data augmentation by learning statistical laws of the input data and generating data samples similar to the input data but not completely repeated [12]. In recent works, GAN and its variants are used in medical image generation. For instance, deep convolutional GAN (DCGAN) is proposed to synthesize realistic prostate disease plaques [13, 14], generate retinal images [15], and synthesize different types of plaques in liver CT [16]. In [17], DCGAN is used to generate high-resolution MR data with only a small number of samples. In 2019, progressive GAN is used to synthesize high-resolution images of skin lesions, which can “cheat” professional dermatologists [18]. Although CT images of lung cancer nodules can be generated by GAN [19], the synthetic lung cancer nodules are indistinguishable from real ones [20], even for radiologists [21]. Evidently, it is still difficult to generate high-resolution CT images of early lung nodules from a small size of labelled samples.

In this work, we developed a method to synthesize quality CT images of early lung nodules using a priori knowledge GAN model from small-size labelled samples. We designed the network to acquire some priori knowledge before executing the generation task. Especially, a knowledge acquisition network and a sharpening network are designed for priori knowledge acquisition, and then, a GAN model is developed to produce CT images of early lung nodules. The contributions of this work are as follows:

- An autoencoder is developed for priori knowledge curation and to retain information on the spatial position, size and shape
- A priori knowledge sharpening layer is embedded to make the model converge quickly

As a result, the CT images generated by SLS-PriGAN are used to train a fast R-CNN network. It achieves a recognition accuracy of 91%, recall rate of 81%, and *F*1 score of 0.85 in identifying clinic CT images of early lung nodules. This provides an effective way of identifying early lung nodules from CT Images generated by deep learning methods with small size samples. It shows that the data enhancement and generation method based on GAN is feasible in alleviating the dilemma caused by the small number of samples.

It is worth noting that the prior knowledge GAN is a problem and domain-specific deep learning algorithm, which is different from the concept of “transfer learning.” Transfer learning uses a pretrained machine learning model for a new but similar problem.

## 2. Method

We herewith propose a GAN-based generative model, named, SLS-PriGAN, to generate high-resolution CT images of early lung nodules. As shown in Figure 1, the main network of our SLS-PriGAN is a stack of GAN networks, which includes a generator, a discriminator, a priori knowledge generation module, and a fusion control module.

The generator accepts a random vector and integrates the output of priori knowledge module to synthesize the image. In image synthesis, a random control module is introduced to achieve the goal of diversification. If the random control module is removed, the generated image will be more inclined to the original image, and the randomness of the generated image will be destroyed. During data simulation, it is found that it is sufficient to use up to 2 random control modules. The discriminator network module reads both pseudo and actual images to analyze and understand their differences and eventually achieve the syntheses.

Incorporating priori knowledge into the generation module is one of the main contributions of SLS-PriGAN, which accelerates the convergence of the model and makes the synthesized image more realistic thus producing more accurate results.

### 2.1. The Generation Network with a Prior Knowledge

During generating process, it uses noise, such as image attributes and categories, to fit feature information. We need to adjust the distribution of high dimensional vectors from low dimensional vectors to synthesize high-resolution CT images, which is a challenge in the case of using small size labelled samples.

The design of the generation network is shown in Figure 2, which includes a knowledge acquisition network and a sharpening network.

The priori knowledge acquisition network is constructed by a convolutional autoencoder (CAE) [22]. The CAE is a structure composed of an encoder and a decoder, and it is trained by the reconstruction loss between the decoded data and the original data [23]. The training process of the CAE is shown in Figure 3. The autoencoder preserves the main features of an image and extract information by encoding and decoding the image.

Let *x* be the input image, *h* be the latent variable, and $\hat{x}$ be the reconstructed image. Ideally, the reconstructed image of the training output should be similar to the original image. The encoder and decoder are represented by Equations (1) and (2), respectively:

(1) $$\begin{array}{c} h=\sigma_{e}\left(W_{1}x+b_{1}\right), \end{array}$$

(2) $$\begin{array}{c} \hat{x}=\sigma_{d}\left(W_{2}h+b_{2}\right), \end{array}$$

where *W*_1_, *b*_1_ are encoding weights and offsets, *W*_2_, *b*_2_ are decoding weights and offsets, and *σ*_*e*_, *σ*_*d*_ are the nonlinear transformations used in the encoding and decoding processes. The convolutional autoencoder uses convolution to linearly transform the input signal and implements a weight sharing strategy. The reconstruction process is a linear combination of basic image blocks that are hidden and coded.

The encoder encodes the input high-dimensional data to obtain the expression of the low-dimensional hidden layer. The decoder decodes the low-dimensional hidden layer to reconstruct the high-dimensional output with the same size as the input. It is further handed over to the lower network to extract and express knowledge. We used variational autoencoders (VAE) in SLS-PriGAN to extract priori knowledge. As shown in Figure 4, after passing through the VAE network, we can directly obtain superficial feature information about shape, size, etc. Our priori knowledge includes information such as the shape and size of the lungs. In addition, high-dimensional and abstract features will be extracted by the neural network.

The knowledge acquisition module further refines the acquired knowledge. Image feature learning is one of the important capabilities of convolutional neural networks (CNN). We access the knowledge sharpening module after acquiring a priori information in order to fully exploit the acquired knowledge features. The sharpening network prevents the collapse of the network. The priori knowledge is further extracted, and the global information of the original image is retained. The priori knowledge module is able to overcome the notorious problems that GAN models often encounter, i.e., difficult to convergence and easy to collapse.

### 2.2. Fusion Control Network

A fusion control module is added to the generator, which implements the additions to the generator's priori knowledge. As well, a random control module is applied to give the generated image a variety and authenticity of detailed information.

#### 2.2.1. Integration of Priori Knowledge

The fusion control network is shown in Figure 5, which includes two parts: the fusion of priori knowledge *W* and the fusion of random noise *N*. As shown in Figure 5, we generally put through the priori knowledge in the 8 × 8 pixel resolution image synthesis process. The intermediate vector *W* is summed with the feature map *S* channel by channel, which realizes the control of the priori knowledge over the body structure of the generated image.

#### 2.2.2. Random Control

The initial random noise input often makes the generated image closer to the real image. We introduced random noises at different locations in the network to make the composite images more diverse. Generally, the lower layers of the network control the high-dimensional information of the generated image, such as the overall structure of the lungs. The relatively high layer tends to control the detailed information of the generated image, such as the information on lung nodules. We added scaled noises to each channel of the generation network at different resolution stages to make the noise only affect the subtle changes in the picture style and then obtain different visual expressions by changing the resolution level.

#### 2.2.3. The Loss Function of the Network

The loss consists of two parts, which are from priori knowledge acquisition module and the generative adversarial network module. The loss can be calculated by Equation (3) [24, 25].

(3) $$\begin{array}{c} \text{Loss}=J_{\text{CAE}}+D_{\text{loss}}+G_{\text{loss}}. \end{array}$$

*D*_loss_ and *G*_loss_ are the loss of discriminator and generator, respectively.

The purpose of the priori knowledge acquisition network is to minimize the error between input *x* and output$\hat{\text{x}}$. Therefore, the loss function that can be used is as follows:

(4) $$\begin{array}{c} J_{\text{CAE}}\left(W\right)=\sum \left(L\left(x,\hat{x}\right)\right)+\lambda {\left\|W\right\|}_{2}^{2}. \end{array}$$

Cross-entropy function *L* is taken as the loss function. The value of parameter *λ* ranges from 0 to 1, which is used to control the weight *W*. Using *λ*, we suppress the influence of static noise, improve the generalization ability of the model, and avoid overfitting. As for the second part, we use Wasserstein Gradient Penalty (WGAN-GP) [26] loss to make the model easy to train, which is as follows:

(5) $$\begin{array}{c} D_{\text{loss}}:E_{x\sim P_{g}}\left[D\left(x\right)\right]-E_{x\sim P_{r}}\left[D\left(x\right)\right]+\lambda E_{x\sim \chi }\left[{\left\|\nabla_{x}D\left(x\right)\right\|}_{p}\right]-1, \end{array}$$

(6) $$\begin{array}{c} G_{\text{loss}}:-E_{x\sim P_{g}}\left[D\left(x\right)\right]. \end{array}$$

## 3. Experiments and Result Discussion

The study was approved by the ethical committee of The Third Hospital of Shandong Province. According to the ethical committee policy, this is a completely anonymous, retrospective study. All sensitive information of the data was removed. The experimental protocols were approved by the hospital, and all methods were carried out per relevant guidelines and regulations.

### 3.1. Training and Testing Dataset

The training and testing dataset of CT images are collected all from The Third Hospital of Shandong Province, China. We curated a total of 673 lung cancer CT images, among which 373 lung cancer CT images are with nodules and selected as the training dataset. The location of the lesion in the CT image is marked by radiologists. The remaining 300 CT images of lung nodules were used as the test set for validation.

### 3.2. Image Synthesis

The structure of the SLS-PriGAN makes model training efficient by introducing a priori knowledge module and a random control module. It does not require redundant techniques hence avoiding possible model collapse. The model has achieved high-quality and high-resolution image generation compared to some work in the current literature, e.g., the method outperformed deep convolutional GAN (DCGAN), see Figure 6.

As shown in Figure 6, at the beginning of training, our SLS-PriGAN showed better fitting ability because of the integration of the priori knowledge. When the training epochs increased gradually, it exhibited a stronger convergence ability. At the epoch of 200, comparing to the DCGAN-generated image with a blurred piece, the synthetic image of the proposed method could be seen as a coarse outline. By epoch 3500, the images synthesized by the proposed method already have a clear lung outline, while DCGAN apparently fell into the trap of image style at epoch 1500 without further convergence.

Figure 7 shows a further qualitative result comparison, which shows that the SLS-PriGAN achieved better results than DCGAN when they were trained for the same number of times. After 47,000 iterations of training, DCGAN-generated images showed structural flaws. The proposed method retained the structural and content accuracy and generated images of higher quality with less significant noise. It is worth mentioning that during the training of DCGAN, the model collapse often occurred, and it was more difficult to synthesize better quality images, yet our network is not prone to such phenomenon. In addition, it is possible for the DCGAN generator to fool the discriminator with images that do not match the lung structure, which is due to the fact that DCGAN uses uncontrolled random noise, but SLS-PriGAN can obviate it.

### 3.3. Experimental Results

It is usually less possible to train an accurate recognition network model using only about 300 images and then recognize the remaining 300 CT images in the test set. With SLS-PriGAN, we generated 4000 CT images to enhance the training set. The generated training set is used to train a general faster R-CNN for lung nodule recognition from CT images. It is shown, in Figure 8, that the results of the performance of the test set with 300 CT images of lung nodules. It achieved the recognizing accuracy of 91%, recall rate of 81%, and *F*1 score of 0.85 in identifying clinic CT images of early lung nodules. The detailed information can be found in Table 1.

Figure 8 shows the qualitative result of early lung nodule detection using Faster R-CNN working on the synthesized data produced by SLS-PriGAN. The four images were randomly selected; the numbers shown in the red labels are the probability of the presence of lung nodules, e.g., 0.93 means that there is a 93% chance of the detected object being a lung nodule.

## 4. Conclusion

In this paper, we propose an SLS-PriGAN model with prior knowledge to generate CT images of early lung nodules from small-size labelled samples. Specifically, a knowledge acquisition network and a sharpening network are designed for priori knowledge learning, and then, a GAN model is developed to produce CT images of early lung nodules. As a result, a general FR-CNN network is trained by the CT images generated SLS-PriGAN, and it achieved a recognizing accuracy of 91%, recall rate of 81%, and *F*1 score of 0.85 in identifying early lung nodules in clinic CT images. This provides a viable way of identifying early lung nodules from CT Images by deep learning with small-size labelled samples. Our study focused on CT images of lung nodules; it is believed that the proposed network model should perform equally well for other problems.

For future research, it is worth investigating the priori knowledge-driven learning strategies, as well as the other kind of cancers of CT images with a small size of labelled samples [27–29], feature-based approaches [30], and a transfer learning enhanced GAN [31].

## Figures and Tables

**Figure 1:** The overall design of SLS-PriGAN.

**Figure 2:** A priori knowledge generation network.

**Figure 3:** The convolutional autoencoder.

**Figure 4:** Our priori knowledge includes information such as the shape and size of the lungs.

**Figure 5:** The details of the fusion control module.

**Figure 6:** The training results of SLS-PriGAN comparing DCGAN, the results of 200, 1500, 2400, and 3500 epochs of training.

**Figure 7:** The generated result comparison with real CT images and DCGAN images.

**Figure 8:** The lung nodule detection of the faster R-CNN on SLS-PriGAN generated images.

**Table 1:** The lung nodule detection results using faster R-CNN on synthesized data generated by SLS-PriGAN and DCGAN.

Train data	Method	Precision	Recall	*F*1
G_dataset1	SLS-PriGAN	0.91	0.81	0.85
G_dataset2	DCGAN	0.88	0.78	0.82
R_dataset	—	0.92	0.90	0.89

G_dataset1 and G_dataset2 are synthesized datasets generated by SLS-PriGAN and DCGAN, respectively. R_dataset is the real CT image data without any modification or synthesized data, which, in this case, can be considered as ground truth to benchmark with two other methods.

## Data Availability

Data are available from the authors upon reasonable request.
